The article "The Potential Role of Matrix Rhythm Therapy in Managing Chronic Low Back Pain: A Scoping Review" was published in 2024. Journal: Cureus.

# The Potential Role of Matrix Rhythm Therapy in Managing Chronic Low Back Pain: A Scoping Review

**DOI:** 10.7759/cureus.72088

**Published:** 2024-10-22

**Authors:** Sumbul Ansari, Kamini Sharma, Zahid Khan

**Affiliations:** 1 Department of Physiotherapy, School of Medical and Allied Health Sciences, Galgotias University, Greater Noida, IND; 2 Department of Physiotherapy, Teerthankar Mahaveer University, Bagadpur, IND; 3 Acute Medicine, Mid and South Essex National Health Service Foundation Trust, Southend-on-Sea, GBR; 4 Cardiology, Barts Heart Centre, London, GBR; 5 Cardiology and General Medicine, Barking, Havering and Redbridge University Hospitals National Health Service Trust, London, GBR; 6 Cardiology, Royal Free Hospital, London, GBR

**Keywords:** disability, functional impairment, marhythe, matrix rhythm therapy, non-pathological chronic low back pain, non-specific chronic low back pain, physical rehabilitation, quality of life, thoracic spinal manipulation, vibromassage

## Abstract

Chronic low back pain (CLBP) is a widespread issue, and matrix rhythm therapy (MRT), a non-invasive therapy using low-frequency vibrations, is gaining interest for CLBP. However, evidence for its effectiveness and safety remains unclear. This scoping review aimed to systematically map and synthesise the existing literature on using MRT to manage CLBP. A comprehensive search of Medical Literature Analysis and Retrieval System Online (MEDLINE), PubMed, Web of Science, Directory of Open Access Journals (DOAJ), and Scopus was conducted for randomised controlled trials (RCTs) published through March 2024. The methodological quality was systematically evaluated using the Physiotherapy Evidence Database Scale (PEDro). The initial search yielded a total of 47 articles. After screening the abstracts and full articles, two studies were included, with a mean score of 5/10 on the PEDro scale. A qualitative review was performed of the two selected RCTs. Meta-analysis was not possible because of the small number of articles in the study. While preliminary findings from the two studies suggest that MRT may be superior to Pilates and combined physical therapy for pain and disability in CLBP, these results require cautious interpretation because of limited research. Further high-quality investigations, particularly well-designed RCTs, are warranted to definitively assess the effectiveness of MRT in managing the pain, function, and other aspects of CLBP.

## Introduction and background

Low back pain (LBP) is caused by discomfort, muscle strain, or stiffness felt in the area between the lower ribs and buttocks, sometimes radiating down the legs [1]. Studies have shown that LBP is a significant health concern [2,3]. The triggering factors of LBP can be identified in only 10-15% of patients, including root compressions, vertebral fractures, tumours, infections, inflammatory diseases, spondylolisthesis, vertebral stenosis, or proclaimed instability [4]. For the remaining 85-90% of patients, identifying the source of pain is challenging, and the term non-specific LBP (NSLBP) is typically used in these cases [5-7]. The duration of pain determines its classification as acute (less than six weeks), subacute (six to 12 weeks), and chronic (> 12 weeks) [8].

The article "The Potential Role of Matrix Rhythm Therapy in Managing Chronic Low Back Pain: A Scoping Review" was published in 2024. Journal: Cureus.

LBP remains the primary contributor to years lived with disability (YLDs) globally. In 2020, over 500 million cases of LBP were documented worldwide [9]. Although age-adjusted rates have shown a modest decline over the past three decades, projections indicate a significant increase, with over 800 million people expected to be afflicted by LBP globally by 2050 [9]. The treatment for LBP, whether medication or therapy, depends on the underlying cause [10]. In terms of management, most studies [2,11-13] recommend non-pharmacological treatments for chronic LBP (CLBP) such as physical activity, physiotherapy, exercise therapy, and education. In some cases, multidisciplinary rehabilitation is recommended as primary treatment. Pharmaceutical therapies, including injections, topical applications, or oral medications, remain contentious but may be available for patients meeting specific criteria.

Individuals with CLBP often lack a precise diagnosis. For most individuals with LBP, non-pharmacological therapies such as physical activity and psychosocial management are preferred. In addition, adjunctive pharmacological therapies may also be used. Surgical and interventional procedures are available for a small subset of individuals who are unresponsive to conventional treatments [14]. Matrix rhythm therapy (MRT) is a dynamic external treatment that was developed by Randoll et al. [15]. It represents a novel approach to managing pain and mobility restrictions and is an electrotherapeutic modality stemming from Randoll's foundational research in Germany [15]. The extracellular matrix is the primary medium through which cellular activities, preventive, therapeutic, regenerative, or destructive, impact the cellular environment.

Research indicates that the human body oscillates at a frequency between 8 and 12 Hz, and a specially designed and authorised Matrixmobil resonator (MaRhyThe-Systems GmbH & Co. KG, Gröbenzell, Germany) generates mechano-magnetic pulsations in the MRT. This method stimulates skeletal muscles within their natural frequency range of 8-12 Hz through mechano-magnetic alternating fields, leading to rhythmic microextension of the muscle tissue. By gently and harmoniously pulsing, MRT helps restore extracellular matrix vibrations, allowing cells to re-establish their natural oscillations. This process enhances the delivery of oxygenated blood and nutrients through the extracellular matrix and facilitates the removal of waste products, acids, and gases [15,16]. This non-invasive therapy is often used to treat wound healing, pain, injuries, and musculoskeletal issues [17]. MRT is indicated for conditions such as tissue oedema, decreased flexibility, muscle spasms, joint hypomobility, and acute or chronic painful muscular and neurological disorders [18].

The article "The Potential Role of Matrix Rhythm Therapy in Managing Chronic Low Back Pain: A Scoping Review" was published in 2024. Journal: Cureus.

MRT supports normal physiological functions, both intracellularly and extracellularly, by maintaining normal tissue pH through micro mobilization with the applicator. Empirical research has shown that increased microcirculation within tissues aids in the elimination of metabolic waste products, reduces oedema, and improves soft tissue extensibility [19,20]. CLBP is a widespread and disabling condition with numerous treatment options, including medications, surgery, physical therapy, and alternative therapies, such as acupuncture. MRT offers a promising, non-invasive option within the realm of physical therapy. However, the specific effects of MRT on CLBP remain relatively unknown. This scoping review aims to address this knowledge gap by examining existing research on MRT for CLBP management.

## Review

Methodology

Eligibility Criteria

To be eligible for inclusion in this review, prospective studies were required to meet specific criteria: randomised controlled trials (RCTs) involving patients diagnosed with CLBP, written in English, and reporting pain and disability as outcomes. Studies employing MRT either as a standalone intervention or in combination with other treatments and comparing outcomes with a control group (placebo, no treatment, or alternative therapy) were considered for inclusion. Articles not presented in full-text format, conference proceedings, grey literature, and abstracts were excluded from this review. No restrictions were placed on the quality rating (as assessed by the Physiotherapy Evidence Database (PEDro) scale score) of the included studies given the limited number of research studies meeting the eligibility criteria. 

Data Sources and Searches

We conducted a comprehensive search of scientific electronic databases including PubMed, Scopus, Directory of Open Access Journals (DOAJ), and Web of Science to identify clinical trials from their inception until March 2, 2024, following the PICO (Populations, Interventions, Comparators, and Outcome) framework [19]. In this review, the PICO framework was operationalised as follows: P: Patients diagnosed with CLBP, I: Interventions involving MRT, C: Control group, and O: Assessment of pain and disability outcomes. The search strategy encompassed the following keywords or combinations: (1) ‘low back pain’, OR ‘back pain’, OR ‘backache’, OR ‘non-specific low back pain’, OR ‘chronic low back pain’, OR ‘non-specific chronic low back pain’; (2) ‘Matrix rhythm therapy’, OR ‘MaRhyThe®’, OR ‘vibromassage’ (3) ‘disability’ and (4) (1) AND (2), (1) AND (2) AND (3) (Table 1). Relevant publications were identified by reviewing the reference lists of the selected articles. 

The article "The Potential Role of Matrix Rhythm Therapy in Managing Chronic Low Back Pain: A Scoping Review" was published in 2024. Journal: Cureus.

**Table 1:** Keywords used for literature search DOAJ: Directory of Open Access Journals

Database	Keywords	Number of results
Scopus	"Chronic low back pain" OR "Low back pain" OR "Back pain" OR "backache" OR "Non-specific low back pain" OR "Non-specific chronic low back pain" AND "Matrix Rhythm Therapy" OR " MaRhyThe®" OR "Vibromassage"	13 results
Web of Science	"Chronic low back pain" OR "Low back pain" OR "Back pain" OR "backache" OR "Non-specific low back pain" OR "Non-specific chronic low back pain" AND "Matrix Rhythm Therapy" OR " MaRhyThe®" OR "Vibromassage"	6 results
PubMed	"Chronic low back pain" OR "Low back pain" OR "Back pain" OR "backache" OR "Non-specific low back pain" OR "Non-specific chronic low back pain" AND "Matrix Rhythm Therapy" OR " MaRhyThe®" OR "Vibromassage"	28 results
DOAJ	"Chronic low back pain" OR "Low back pain" OR "Back pain" OR "backache" OR "Non-specific low back pain" OR "Non-specific chronic low back pain" AND "Matrix Rhythm Therapy" OR " MaRhyThe®" OR "Vibromassage"	0 results

Data Extraction and Synthesis

Two authors independently screened and selected RCTs according to the predetermined eligibility criteria. Subsequently, the authors manually extracted the data using an Excel spreadsheet (Microsoft Corporation, Redmond, Washington, United States). Following data extraction, the third author verified the accuracy of the extracted data. The extracted data included authors' names, year of publication, study design, participant characteristics (e.g. sample size, sex distribution, and age), inclusion and exclusion criteria, details of the interventions (including number of groups, treatment frequency, and duration), variables assessed (e.g. pain and disability), and study results. 

Methodological Quality Assessment

Two authors assessed the methodological quality of the papers using the 11-point PEDro scale (Table 2) [21,22]. Discrepancies in assessments were resolved either by a third author or through discussion to reach a consensus. The PEDro scale incorporates elements from the Jadad scale and the Delphi list [23,24] and comprises 11 items, each answered with either ‘yes’ or ‘no’. A score of ‘1’ is assigned for each present item, while ‘0’ is given if absent. Notably, the item ‘eligibility criteria were specified’ is excluded from the final score calculation. Study quality was categorised as poor, fair, good, or excellent based on PEDro scores < 4, 4-5, 6-8, or 9-10, respectively [24,25]. The risk of bias (RoB-2) tool was used to assess studies for risk of bias assessment (Figures 1, 2).

The article "The Potential Role of Matrix Rhythm Therapy in Managing Chronic Low Back Pain: A Scoping Review" was published in 2024. Journal: Cureus.

**Table 2:** Methodological quality rating of all the selected studies based on the PEDro scale Physiotherapy Evidence Database (PEDro) scale

Criterion	Gohil et al., 2023 [26]	Ozcan et al., 2021 [27]
Eligibility criteria were specified	Yes	Yes
Subjects were randomly allocated to groups (in a crossover study, subjects were randomly allocated an order in which treatments were received)	Yes	Yes
Allocation was concealed	No	No
The groups were similar at baseline regarding the most important prognostic indicators	No	Yes
There was blinding of all subjects	No	No
There was blinding of all therapists who administered the therapy	No	No
There was blinding of all assessors who measured at least one key outcome	No	No
Measures of at least one key outcome were obtained from more than 85% of the subjects initially allocated to groups	Yes	Yes
All subjects for whom outcome measures were available received the treatment or control condition as allocated or, where this was not the case, data for at least one key outcome was analyzed by “intention to treat”	Yes	Yes
The results of between-group statistical comparisons are reported for at least one key outcome	Yes	Yes
The study provides both point measures and measures of variability for at least one key outcome	No	Yes
Total points (out of 10)	4	6

**Figure 1:** Risk of bias (RoB) traffic light chart for studies including in the scoping review

**Figure 2:** Summary plot for risk of bias (RoB) plot for studies included in the scoping review

Results

The Preferred Reporting Items for Systematic Reviews and Meta-Analyses (PRISMA) flow diagram shows the selection process of the included studies and literature search (Figure 3). An initial search across diverse electronic databases and supplementary sources yielded 47 articles, with the following distribution: 13 from Scopus, 6 from Web of Science, 0 from DOAJ, and 28 from PubMed. Upon the removal of duplicates, a careful screening of titles and abstracts was conducted for the remaining 43 articles. Subsequently, three articles underwent full-text assessment for eligibility. Of these, one article was excluded because of full-text unavailability [26]. Consequently, two articles meeting all the inclusion criteria were identified for detailed analysis [27,28]. 

The article "The Potential Role of Matrix Rhythm Therapy in Managing Chronic Low Back Pain: A Scoping Review" was published in 2024. Journal: Cureus.

**Figure 3:** PRISMA 2020 flow diagram showing literature and selection PRISMA: Preferred Reporting Items for Systematic Reviews and Meta-Analyses

Across the final two RCTs, a combined total of 82 individuals with CLBP were enrolled. Sex distribution varied among the studies, with one study not reporting the sex of the participants and the other study involving both male and female patients [27,28]. Among the 82 participants enrolled in the two RCTs, 17.07% were male, 21.95% were female, and 60.97% remained unspecified. The age of the participants in these two trials ranged from 18 to 50 years. The characteristics of the included studies are summarised in Table 3.

**Table 3:** Summary of the included studies RCT: Randomized controlled trials; N: Total number of participants; CLBP: Chronic low back pain; HP: Hot pack; US: Ultrasound; TENS: Transcutaneous electrical nerve stimulation; MRT: Matrix rhythm therapy; MPQ: McGill pain questionnaire; ODI: Oswestry disability index; SF-36: Short form-36; NR: Not reported; NPRS: Numeric pain rating scale

Author	Study design	Participants	Inclusion (I) and exclusion (E)	Treatment	Variables	Effect and results
Gohil et al., 2023 [27]	RCT	N=50, Age: 18-35	I = Age: 18-35 years with CLBP; E = All other patients	Group A: MRT (45 minutes for three sessions per week for two weeks). Group B: Pilates (45 minutes for three sessions per week for two weeks) (warm-up + 18 different core muscle exercises+ cool-down).	Pain (NPRS), Lumbar spine mobility (modified Schober’s test), Pelvic inclination (inclinometer), Functional impairment (ODI)	A post-intervention significant improvement (p<0.05) was seen in Groups A and B. There was a statistically significant difference between the groups for all variables (p<0.05).
Ozcan et al., 2021 [28]	RCT	N=36, (Male=14, Female=18) Age: 36.41 ±8.91	I = Age between 20-50 years, diagnosed with CLBP, and volunteered to participate; E = previous spinal surgery, neurological losses due to free fragment and/or disc herniation, spinal instability, severe systemic disease (cardiovascular, metabolic, pulmonary, and malignancy), pregnancy or at least one year postpartum, diagnosed psychiatric problem, and receiving pharmacological treatment for pain	Experimental group: Combined physiotherapy program (HP, US, and TENS) + training to protect during daily life activities (avoiding sudden movements, protection against cold, not lifting heavy loads, among others) and an exercise program (strengthening, stretching, range of motion, and posture exercises) to be implemented at home + informed about nutrition, sleep patterns, and energy-saving + MRT. Control Group: Combined physiotherapy program (HP, US, and TENS) + training to protect during daily life activities (avoiding sudden movements, protection against cold, not lifting heavy loads, among others) and an exercise program (strengthening, stretching, range of motion, and posture exercises) to be implemented at home + informed about nutrition, sleep patterns, and energy-saving.	Pain (MPQ), Disability levels (ODI), Quality of life (SF-36)	In the experimental group, a statistically significant difference was found in total pain level, disability level, and all subdimensions except the ‘‘Emotional Role’’ subdimension of Short Form 36 (SF-36) and total SF-36 scores (p<0.05). In the control group, statistically significant differences were found in disability level, the ‘‘Vitality’’ and ‘‘Bodily Pain’’ subdimensions of SF-36, and total SF-36 scores (p<0.05).

Quality Assessment

The methodological quality of articles was assessed using the PEDro scale. One study [27] was classified as poor-quality (4/10) on the PEDro scale, whereas the other study [28] was classified as good-quality (6/10) (Table 2). These classifications were based on established cut-off scores, as referenced in previous studies [21]. The mean PEDro score across all included studies was 5, indicating an overall fair quality of the two studies.

The article "The Potential Role of Matrix Rhythm Therapy in Managing Chronic Low Back Pain: A Scoping Review" was published in 2024. Journal: Cureus.

Interventions

Gohil et al. administered MRT for 45 minutes across three sessions for the experimental group and Pilates for 45 minutes across three sessions per week for two weeks for the control group (Table 2). Ozcan et al. introduced an intervention that combined MRT with a comprehensive physiotherapy program. This program involved applying a hot pack for 20 minutes to provide superficial heating to the lumbar and upper sacral area, followed by ultrasound treatment for five minutes with an intensity of 1.5 watts/cm2 and a frequency of 1 MHz. Additionally, conventional transcutaneous electrical nerve stimulation (TENS) was administered for 20 minutes, utilising a frequency of 100 Hz and a duration of 50 ms to alleviate pain. This intervention was provided to the intervention group, whereas the control group received a combined physiotherapy program without MRT. Both groups underwent these interventions five days a week (weekdays) for a total of 10 sessions over two weeks (Table 3). Gohil et al. reported that MRT is effective in several musculoskeletal conditions. In the study by Ozcan et al, a significant difference in total pain and disability level was observed in the intervention group receiving MRT, whereas the control group receiving physiotherapy only had a significant improvement in the disability level. These two studies demonstrated that the combined physiotherapy and matrix rhythm intervention therapy program had a peculiar effect on pain, disability level, and quality of life in patients with CLBP. 

The article "The Potential Role of Matrix Rhythm Therapy in Managing Chronic Low Back Pain: A Scoping Review" was published in 2024. Journal: Cureus.

Outcome Measures 

Both RCTs examined the pain and disability outcomes. Gohil et al. (2023) used the numeric pain rating scale (NPRS) for pain and the Oswestry disability index (ODI) for disability assessment [27]. Ozcan et al. (2021) used the McGill Pain Questionnaire (MPQ) for pain and the ODI for disability [28]. Other outcomes assessed included quality of life (Short Form-36 (SF-36)) [28], lumbar spine mobility (modified Schober’s test) [27], and pelvic inclination (inclinometer) [28]. 

A Qualitative Synthesis of the Interventions 

According to the findings of Ozcan et al.'s study (2021), a statistically significant between-group difference was observed solely in the ‘general health perceptions’ subdimension of SF-36, favouring the intervention group (Table 2) [28]. Upon examining the effect sizes within each group, it was noted that the MRT program combined with physiotherapy exhibited moderate to high effectiveness in the intervention group, whereas the combined physiotherapy program alone in the control group demonstrated a slight to moderate level of effectiveness [28]. The findings of the study by Gohil et al. (2023) showed that MRT demonstrated notably substantial improvements in pain, lumbar flexibility, functional impairments, and pelvic inclination when compared to Pilates in individuals with CLBP [27].

Discussion 

This investigation marks, to the best of our knowledge, the first systematic amalgamation of research concerning the effects of MRT on pain and disability in patients with CLBP. This domain appears to be a burgeoning area with substantial clinical potential. The current systematic review involved meticulous extraction, critical appraisal, and the synthesis of extant evidence. The present critical evaluation and synthesis of studies indicate superior outcomes associated with MRT compared with interventions administered to the control groups. Nevertheless, caution is required in the interpretation of findings owing to the constrained quantity (only two) of studies and the heterogeneity observed among the included studies. 

This review identified only two studies meeting the inclusion criteria, highlighting the limited research on MRT for CLBP management. Notably, none of the included studies defined CLBP according to their inclusion criteria [27,28]. This highlights the importance of adapting standardised CLBP definitions for patient recruitment to ensure consistency and generalisability across studies. Both studies implemented a two-week intervention, but the frequency differed [27,28]. Gohil et al. (2023) delivered MRT three times a week, while Ozcan et al. used it five times weekly. Notably, these studies diverged in their treatment approaches. Gohil et al. employed MRT as the sole intervention, while Ozcan et al, combined MRT with physical therapy, suggesting MRT as an adjunct treatment in their study [27, 28].

The article "The Potential Role of Matrix Rhythm Therapy in Managing Chronic Low Back Pain: A Scoping Review" was published in 2024. Journal: Cureus.

Gohil et al. conducted a study with methodological limitations that compromise its quality. The allocation of participants into groups was not concealed, raising concerns about potential selection bias. Additionally, the authors did not report whether the groups were similar at baseline in terms of the important prognostic factors. Furthermore, there was no blinding of participants, assessors, or therapists, which could have introduced bias due to expectations. Finally, the results section lacked the reporting of both point estimates and variability measures for at least one key outcome. These shortcomings collectively classify the study as having poor quality according to the established criteria [25]. In contrast, Ozcan et al. also lacked concealed allocation and blinding of participants, assessors, and therapists. However, despite these limitations, the study might be considered to have good overall quality based on other criteria of the PEDro scale [25]. Despite these noteworthy limitations, significant improvements were observed in pain and disability after the intervention in both studies [27,28]. However, greater changes in pain and disability were observed in the group that received MRT. The potential mechanism(s) underlying these improvements could be attributed to physiological processes associated with MRT. MRT applies external oscillatory forces to synchronise the vibrations of muscle cells. The proposed mechanism involves an MRT device that induces vibrations in the extracellular matrix fluid that surrounds the muscle cells. This, in theory, resonates with the natural contractile oscillations of muscle fibres, potentially enhancing blood flow within skeletal muscles [16]. Increased microcirculation within tissues aids in the elimination of metabolic waste products, reduces oedema, and improves soft tissue extensibility [19], thus plausibly reducing pain. Due to the limited research in this area, definitive conclusions cannot currently be drawn regarding the effectiveness of MRT in reducing pain and disability in individuals with CLBP. Future high-quality RCTs are required to investigate this potential application.

Several systematic reviews and meta-analyses have evaluated the efficacy of various interventions for CLBP [29,30]. While the findings of these studies are diverse, there is a growing interest in exploring novel treatment options, such as MRT. Pain and disability assessments are critical patient-reported outcomes that should be consistently evaluated in future studies. Gianola et al. performed a meta-analysis by including 8765 participants from 46 trials [29]. This study showed that manual therapy significantly reduced pain symptoms in patients compared with inert treatment, and in terms of disability, pharmacological therapy and muscle relaxants were statistically significant compared with inert treatment. Wallwork et al. performed a meta-analysis by including 95 studies, with 60 separate cohorts in the systematic review including 17974 patients and 47 cohorts including 9224 patients in the meta-analysis. This study showed that patients' lower back shows improvement in the first six weeks; however, patients tend to have ongoing pain and disability despite the initial improvement [30].

The article "The Potential Role of Matrix Rhythm Therapy in Managing Chronic Low Back Pain: A Scoping Review" was published in 2024. Journal: Cureus.

This review provides a valuable analysis of the existing literature on MRT for CLBP. However, with only two studies included, it is essential to conduct further high-quality research to establish definitive conclusions regarding its effectiveness. Future studies should prioritise larger sample sizes, standardised interventions, and rigorous blinding procedures to enhance the reliability and generalisability of the findings. Additionally, investigating the long-term effects of MRT is crucial to understanding its sustained benefits. Comparing the cost-effectiveness of MRT with other CLBP treatments can inform healthcare decision-making. Given the limited number of studies, a meta-analysis was not feasible in this review. Future studies with a larger pool of eligible studies will enable a more comprehensive meta-analysis to provide a stronger evidence base for MRT's effectiveness in managing CLBP.

Strengths and Limitations 

To the best of our knowledge, this is the first systematic review based on RCTs assessing the efficacy of MRT. The main limitation of this study is the limited number of RCTs involved in this study. Further RCTs involving large numbers of patients would be useful to investigate the efficacy of MRT in CLBP.

## Conclusions

The management of CLBP through MRT appears to be a relatively underexplored area, with only three studies identified to date. This current review shows that MRT therapy and combined physiotherapy programs improve patients' quality of life and reduce their pain and disability levels. While two of these studies suggested that MRT might be superior to Pilates and combined physical therapy in reducing pain and disability in CLBP patients, these findings require cautious interpretation due to the limited research available. However, MRT shows considerable promise, particularly considering the ongoing search for optimal CLBP treatments. Preliminary evidence suggests that MRT is a promising intervention strategy. However, high-quality RCTs are necessary to definitively assess its effectiveness. These trials should meticulously evaluate the effect of MRT on pain levels, functional disability, and other subjective and objective parameters. This comprehensive evaluation will help to elucidate the potential role of MRT in managing CLBP.
